# Theoretical Background to Automated Diagnosing of Oral Leukoplakia: A Preliminary Report

**DOI:** 10.1155/2020/8831161

**Published:** 2020-09-13

**Authors:** Kamil Jurczyszyn, Tomasz Gedrange, Marcin Kozakiewicz

**Affiliations:** ^1^Department of Oral Surgery, Medical University in Wrocław, Wrocław, Poland; ^2^Department of Orthodontics, TU Dresden, Dresden, Germany; ^3^Department of Maxillofacial Surgery, Faculty of Military Medicine, Medical University of Lodz, Łódź, Poland

## Abstract

Oral leukoplakia represents the most common oral potentially malignant disorder, so early diagnosis of leukoplakia is important. The aim of this study is to propose an effective texture analysis algorithm for oral leukoplakia diagnosis. Thirty-five patients affected by leukoplakia were included in this study. Intraoral photography of normal oral mucosa and leukoplakia were taken and processed for texture analysis. Two features of texture, run length matrix and co-occurrence matrix, were analyzed. Difference was checked by ANOVA. Factor analysis and classification by the artificial neural network were performed. Results revealed easy possible differentiation leukoplakia from normal mucosa (*p* < 0.05). Neural network discrimination shows full leukoplakia recognition (sensitivity 100%) and specificity 97%. This objective analysis in the neural network revealed that involving 3 textural features into optical analysis of the oral mucosa leads to proper diagnosis of leukoplakia. Application of texture analysis for leukoplakia is a promising diagnostic method.

## 1. Introduction

Oral leukoplakia represents the most common oral potentially malignant disorder [1]. It is a white patch or plaque that cannot be characterized clinically or pathologically as any other disease. It is a classical definition of leukoplakia presented by the World Health Organization. Etiology of leukoplakia is multifactorial. Most important factors are alcohol, smoking cigarettes, poor oral hygiene, electrogalvanic currents, and spicy food irritating oral mucosa. Possibility of malignant transformation of leukoplakia is in the range between 0.2% and 5% [2]. Due to the risk of malignant transformation, it is important to take a proper diagnosis. The golden standard of diagnosis is still histopathological examination, but invasiveness is a main disadvantage of that examination. Fluorescence or autofluorescence of lesions are used in some of the diagnostic systems, such as ViziLite®, ViziLite®PLUS, VELscope®, Identafi®, and Orascoptic DK [3, 4]. The huge wave of electrooptical devices is a base for alterations in oncological prophylaxis in oral squamous cell cancer. There are simple analogous apparatus, such as VELscope and Microlux, which utilize fluorescence or led light. Unfortunately their specificity is very low.

Digital images are consisted of pixels. Pixels build patterns which create texture. Mathematical and statistical analysis of texture patterns is known as texture analysis (TA). Methods of TA are based upon the mathematical analysis of the matrix that represents the distribution of pixel brightness within the image. Texture analysis may be divided into four methods: statistical, structural, model-based, and transform [5, 6]. TA is commonly used in medicine to analyze X-ray photos, computed tomography images, or magnetic resonance images. Intraoral digital photos of leukoplakia seem to be a good material for texture analysis, which will be helpful in early diagnostic.

On the one hand, nowadays, intraoral macrophotography with a digital single lens camera or compact system camera is popular in dentistry. On the other hand, endoscoping image acquisition is possible in oral cavity by maxillofacial surgeons, ENT doctors, or gastroenterologists too. Previously mentioned methods may be the potential source of images which can be analyzed using TA.

Electronic, tele-, and automated diagnosing is possible in the decade when each physician possess a smartphone. Proper small cameras and LED light are in all telephones, and many electrooptical devices are available in dental or medical centers. The minor development is noted in the field of specialized software.

The aim of this study was to create a base of the remote diagnosis system of oral leukoplakia.

## 2. Materials and Methods

### 2.1. Patients

Thirty-five patients affected by leukoplakia were included into this study. All lesions were histopathologically verified (with standard hematoxylin and eosin staining) after taking the specimen from pathologically changed oral mucosa under local anesthesia. The mean age of the study group was 58 years. Exclusion criteria was a high grade dysplasia.

Intraoral photography of normal oral mucosa and leukoplakia was taken using a Canon EOS 500D (Canon, Ōta, Tokyo, Japan) digital camera with a macro ring 13 mm, 50 mm, f1.8 lens (Canon, Ōta, Tokyo, Japan) and ring flashlight YN-14EX (YONGNUO Photographic Equipment, Longhua District, Shenzhen, China). All photos were taken from the same distance (focus distance was locked to achieve it), and optical axis of lens was perpendicular to examined lesion. A polarized filter on the camera lens was applied to reduce any reflections. Directly before taking photo, affected mucosa was getting dry to decrease the risk of reflections.

All procedures were conducted after obtaining the approval of the Ethics Committee of Wroclaw Medical University, Poland (approval No. KB-367/2014).

### 2.2. Image Preprocessing

All of graphical operations were performed in GIMP version 2.10.8 (GNU Image Manipulation Program, https://www.gimp.org/). In the center of the lesion, the region of interest (ROI) with 300 × 300 pixels was selected. Leukoplakia ROI was selected at the center of the lesion, without reference healthy mucosa. Reference mucosa ROI was selected from the same region, for example, if lesion was at the tongue, reference ROI was selected at the tongue. Such prepared fragment of image was cut-off from the original photo. To achieve maximum possible contrast of photography, a high-pass filter was applied. After that, level tools were used to equalize image histogram (to unify contrast of all images). Next, images were converted into the 4 bits grey scale. File was saved into TIFF format without any compression algorithms. All graphical operations are shown in Figure 1. The region of interest was chosen without any visible reflections in all of cases.

### 2.3. Texture Analysis

Optical images (300 × 300 pixels) from 35 cases were transformed to the 4 bit grey scale graphical files imported in MaZda 4.6 (Technical University of Lodz, Poland) software, and texture analysis was performed (Figure 2) [7, 8]. Six textural features were selected: two of run length matrix (long run emphasis inverse moments and short run emphasis inverse moments), two of co-occurrence matrix (entropy as shown in Figure 3 and difference entropy calculated in distance of 5 pixels), and two of Haar wavelet transformation (wavelet energy after a two-dimensional low-pass filter and scale 5 and scale 6 of the transformation) [9–11].

Let *p* (*i*, *j*) be the number of times there is a run of length *j* having grey level *i*. Let *N*_*g*_ be the number of grey levels, and *N*_*r*_ be the number of runs [12]. Definitions of the parameters of the run length matrix *p* (*i*, *j*) are given below.

  Long run emphasis inverse moments:

(1) $$\begin{array}{c} \text{LngREmph}=\frac{\sum_{i=1}^{N_{g}}\sum_{j=1}^{N_{r}}j^{2}p\left(i,j\right)}{C}. \end{array}$$

  Short run emphasis inverse moments:

(2) $$\begin{array}{c} \text{ShrtREmph}=\frac{\sum_{i=1}^{N_{g}}\sum_{j=1}^{N_{r}}p\left(i,j\right)/j^{2}}{C}, \end{array}$$

where the coefficient *C* is defined as

(3) $$\begin{array}{c} C=\sum_{i=1}^{N_{g}}\sum_{j=1}^{N_{r}}p\left(i,j\right). \end{array}$$

The co-occurrence matrix-derived parameters are defined by the equations that follow, where *μ*_*x*_, *μ*_*y*_, and *σ*_*x*_ and *σ*_*y*_ denote the mean and standard deviations of the row and column sums of the co-occurrence matrix, respectively, which are related to the marginal distributions *p*_*x*_(*i*) and *p*_*y*_(*j*).

  Entropy:

(4) $$\begin{array}{c} \text{Entropy}=-\sum_{i=1}^{N_{g}}\sum_{j=1}^{N_{g}}p\left(i,j\right)\log\left(p\left(i,j\right)\right). \end{array}$$

  Difference entropy:

(5) $$\begin{array}{c} \text{DifEntrp}=-\sum_{i=1}^{N_{g}}p_{x-y}\left(i\right)\log\left(p_{x-y}\left(i\right)\right). \end{array}$$

For discrete Haar wavelet transformation, the calculation of energy for frequency 2D subband after passing a low-pass filter (*L*) in scales 5 and 6 was performed:

(6) $$\begin{array}{c} E_{\text{subband},\text{scale}}=\frac{\sum_{x,y\in \text{ROI}}{\left(d_{x,y}^{\text{subband}}\right)}^{2}}{n}, \end{array}$$

where *d* is the wavelet coefficient, and *n* is the number of pixels in region of interest (ROI, i.e., whole image presented in Figure 3 in the upper raw), both at 5^th^ and 6^th^ scales and subband LL. ROIs are reduced in successive scales in order to correspond to subband image dimensions. Output of this procedure is a vector of features containing energies of wavelet coefficients calculated in subband LL at 5^th^ and 6^th^ scales.

ANOVA was performed in Statgraphics Centurion XVI software. Next, procedure uses a probabilistic neural network (PNN in Statgraphics Centurion XVI software) to classify cases into different diagnosis, based on 3 input variables (input factors were the strong distractors of this image analysis: short run emphasis inverse moments, entropy, and wavelet transformation energy in scale 5 of the 35 cases (Figure 4).

### 2.4. Statistical Analysis

The Shapiro–Wilk test was applied to checking normality. One-way analysis of variance (ANOVA) was applied. The difference was considered as significant if *p* < 0.05. Statgraphics Centurion 18 ver.18.1.12 (StarPoint Technologies, Inc., Virginia, USA).

## 3. Results

Summary statistics of selected textural features of oral mucosa are presented in Table 1. Frequency of short run emphasis inverse moments artifacts decreases significantly in leukoplakia lesion (*p* < 0.005). Both methods of calculation of the entropy reveals their decrease in pathology (difference entropy *p* < 0.005 and entropy *p* < 0.001, Figure 5). The superimposition on texture pattern is the highest (the energy is the highest) as far as Haar wavelet transformation considered in scales 5 and 6.

Neural network discrimination shows (Figure 6) full leukoplakia recognition (sensitivity 100%) and specificity 97%. All of leukoplakia images were described properly, and one normal mucosa image was classified as pathological lesion.

## 4. Discussion

Sambandham et al. applied the ViziLite system in case of leukoplakia diagnosis. Their study shows that sensitivity and specificity of ViziLite is about 77.3% and 27.8%, respectively [13]. McIntosh et al. revealed that the Microlux/DL system showed a sensitivity of 77.8% and a specificity of 70.7% in case of leukoplakia diagnosis [14]. Ibrahim et al. revealed that even adding toluidine blue dye did not improve the effectiveness of the Microlux/DL system. At the same study, they showed that the sensitivity was 100% and specificity was 32.4% of Microlux/DL for visualization of suspicious premalignant lesions when considering biopsy as a golden standard [15].

Lalla et al. confirmed that it is possible to detect oral epithelial dysplasia using reflectance spectroscopy (Identafi and DentalEZ). Their study showed that Identafi's system under violet light offered a sensitivity of 12.5% and specificity of 85.4% for detection of oral epithelial dysplasia. It is important to know that high level of clinical experience is required to interpret the results of autofluorescence examination [16].

Chan et al. used texture analysis in case of microcalcifications detection on mammograms. Their result indicates that computerized texture analysis can extract mammographic information that is not apparent by visual inspection. These studies reveal that the level of specificity was 39% and the sensitivity level was 100% [17]. Our results were the same at the level of sensitivity but much higher in aspect of specificity (97%). Li et al. studies confirmed too that mammographic texture analysis was a reliable technique for differential diagnosis of benign and malignant breast tumors. Furthermore, the combination of imaging-based diagnosis and texture analysis can significantly improve diagnostic performance [18].

Short run length emphasis inverse moments detect short lines of pixels which have similar lightness. Their presence in mucosal image is the normal status. As the short lines disappeared, the leukoplakia develops. Similarly, entropy and difference entropy indicate the regions where the fine nest of mucosal surface texture exists. In pathological lesion, that fine texture disappears transforming into white regions, i.e., leukoplakia areas. Haar wavelet transformation results indicate that the pathological lesions of leukoplakia are quite extended due to a significant scale of wavelet transformation (scale 5 and scale 6), which can be superimposed on the pathological texture. That again points that the oral mucosa lost its physiological fine textural appearance.

That objective analysis in the neural network revealed that involving 3 textural features into optical analysis of the oral mucosa leads to proper diagnosis of leukoplakia. One normal sample of oral mucosa was recognized as pathology probably due to subclinical development of pathology in mucous membrane.

The proposed 5 or less features of oral mucosa texture observed in natural or artificial light can be used for developing simple application for a smartphone to significantly improve possibility of oral mucosa leukoplakia.

## 5. Conclusions

Application of texture analysis for oral leukoplakia versus healthy mucosa is a promising diagnostic method, which may be a base of the remote and semiautomatic diagnosis system.

## Figures and Tables

**Figure 1:** Graphical operations of source intraoral photography of leukoplakia.

**Figure 2:** Texture analysis in MaZda. Red region of interest indicates image of oral mucosa leukoplakia. Green region of interest indicates normal oral mucosa. Analyzed images were grey scale 4 bit. RLM, run length matrix features. COM, co-occurance matrix features were calculated on between-pixel distance of 5.

**Figure 3:** Analyzed images. Left column: leukoplakia of oral mucosa. Right column: normal oral mucosa. In top: raw photographic images. In second row: images after transformation to the 8 bit normalized grey scale. Third row: short run emphasis inverse moments map (number of short lines of similar pixels increased in some regions of leukoplakia-left image). In bottom: maps of entropy distribution in the image (inside leukoplakia, foci are dark areas of low entropy mixed with high entropy plates; in normal mucosa, entropy is distributed regularly).

**Figure 4:** Schema of the probabilistic neural network used for discrimination the leukoplakia lesion from normal mucosa.

**Figure 5:** Measured entropy of image of oral leukoplakia (+mean value; | median value). Normal mucosa has more chaotic texture, i.e., higher entropy, than leukoplakia, in which texture is organized in plates (*p* < 0.001).

**Figure 6:** Results of effective discrimination of oral mucosa images (97% of specificity and 100% sensitivity).

**Table 1:** Summary statistics of textural features in normal oral mucosa and leukoplakia lesions.

Textural feature	Reference mucosa	Leukoplakia lesion	ANOVA

Long run emphasis inverse moments	9.70 ± 15.38^*∗*^	13.93 ± 8.90	*F* = 1.99; *p*=0.16
Short run emphasis inverse moments	0.64 ± 0.14^*∗*^	0.56 ± 0.08	*F* = 10; *p* < 0.005
Entropy	1.73 ± 0.12	1.62 ± 0.10	*F* = 16; *p* < 0.001
Difference entropy	0.56 ± 0.09	0.50 ± 0.07	*F* = 11; *p* < 0.005
Wavelet transformation energy LL scale 5	57.44 ± 2.61	67.75 ± 1.52	*F* = 462; *p* < 0.0001
Wavelet transformation energy LL scale 6	56.12 ± 2.61	65.65 ± 1.86	*F* = 309; *p* < 0.0001

^*∗*^Lack of normal distribution.

## Data Availability

The data that support the findings of this study are available from the corresponding author upon reasonable request.
